# The Changing Trend of Paediatric Emergency Department Visits in Malaysia Following the COVID-19 Pandemic

**DOI:** 10.7759/cureus.36512

**Published:** 2023-03-22

**Authors:** Afiqah Syamimi Masrani, Nik Rosmawati Nik Husain, Kamarul Imran Musa, Paula Moraga, Mohd Tahir Ismail

**Affiliations:** 1 Department of Community Medicine, School of Medical Sciences, Universiti Sains Malaysia, Kota Bharu, MYS; 2 Division of Computer, Electrical and Mathematical Science and Engineering, King Abdullah University of Science and Technology, Thuwal, SAU; 3 School of Mathematical Sciences, Universiti Sains Malaysia, Pulau Pinang, MYS

**Keywords:** time series, changepoint analysis, movement control order, covid-19, paediatric, emergency department

## Abstract

Background

The coronavirus disease 2019 (COVID-19) pandemic has impacted the emergency department (ED) due to the surge in medical demand and changes in the characteristics of paediatric visits. Additionally, the trend for paediatric ED visits has decreased globally, secondary to implementing lockdowns to stop the spread of COVID-19. We aim to study the trend and characteristics of paediatric ED visits following Malaysia’s primary timeline of the COVID-19 pandemic.

Methods and materials

A five-year time series observational study of paediatric ED patients from two tertiary hospitals in Malaysia was conducted from March 17, 2017 (week 11 2017) to March 17, 2022 (week 12 2022). Aggregated weekly data were analysed using R statistical software version 4.2.2 (R Foundation for Statistical Computing, Vienna, Austria) against significant events during the COVID-19 pandemic to detect influential changepoints in the trend. The data collected were the number of ED visits, triage severity, visit outcomes and ED discharge diagnosis.

Results

Overall, 175,737 paediatric ED visits were recorded with a median age of three years and predominantly males (56.8%). A 57.57% (p<0.00) reduction in the average weekly ED visits was observed during the Movement Control Order (MCO) period. Despite the increase in the proportion of urgent (odds ratio (OR): 1.23, p<0.00) and emergent or life-threatening (OR: 1.79, p<0.00) cases, the proportion of admissions decreased. Whilst the changepoints during the MCO indicated a rise in respiratory, fever or other infectious diseases, or gastrointestinal conditions, diagnosis of complications originating from the perinatal period declined from July 19, 2021 (week 29 2021).

Conclusion

The incongruent change in disease severity and hospital admission reflects the potential effects of the healthcare system reform and socioeconomic impact as the pandemic evolves. Future studies on parental motivation to seek emergency medical attention may provide insight into the timing and choice of healthcare service utilisation.

## Introduction

Coronavirus disease 2019 (COVID-19) is an infectious disease caused by the SARS-CoV-2 virus. It was first identified in Wuhan, China, and subsequently spread globally. With nearly 400 million confirmed cases and more than five million deaths, the World Health Organization declared the COVID-19 pandemic in March 2020. Health systems worldwide responded by implementing statewide lockdowns to control the pandemic and flatten the epidemiological curve, thus allowing time for the health system to respond [1].

The Ministry of Health Malaysia initiated a COVID-19 preparedness plan in early January 2020, encompassing areas in public health, clinical management and laboratory capacity. Following the exponential rise in locally transmitted COVID-19 cases, Malaysia entered a nationwide lockdown on March 18, 2020. The lockdown, known as the Movement Control Order (MCO), was enforced under the Control and Prevention of Infectious Diseases Act of 1988 and the Police Act of 1967 and defined the following: the complete restriction of movement and social gathering nationwide, a total ban of international travel of all Malaysian citizens or foreign visitors and tourists, the closure of all educational facilities and the closure of all government and private premises, except those involved in essential services. The MCO was lifted in phases and was fully lifted on January 3, 2022, when Malaysia achieved an average number of COVID-19 cases per day below 500, a stabilised public healthcare service with an adequate level of ICU bed usage rate and vaccination coverage of 60% of the population with at least two doses of the COVID-19 vaccine.

The emergency department (ED) is the point of contact for the community for emergency health services. Children below 18 years old make up nearly 35% of the total ED visit worldwide annually, with approximately 15 out of 100 children visiting the ED at least once a year [2-6]. Out of this, more than 40% of paediatric ED visits were children under five years old, most of them being discharged from the ED with a ratio of one hospital admission out of every 14-20 ED visits [2]. Injury and poisoning contribute to the highest proportion of ED visits among children, followed by respiratory disorders, nervous system disorders and infectious diseases [7].

Paediatric ED visits declined following the COVID-19 pandemic in various locations globally. A study of 11 Canadian hospitals has shown a reduction in the total paediatric ED visits during the early phases of the pandemic [8]. A similar finding was observed in Korea, where a 58.1% (95% confidence interval (CI): 57.2%-58.9%, p<0.001) decrease in paediatric ED visits was observed [9]. Despite the decline in number, the proportion of emergent cases, which are conditions that are a potential threat to life, limb or function requiring rapid medical intervention, was almost equal (odds ratio (OR): 1.03, 95% CI: 1.00-1.07, p=0.04) during the early pandemic phases and in the pre-pandemic period [8]. Therefore, we hypothesised that changes in paediatric ED visits have also occurred in Malaysia. We aim to study any changes in the trend and characteristics of paediatric ED visits following the primary timeline of the COVID-19 pandemic in Malaysia.

## Materials and methods

Design and setting

Our time series study consisted of weekly aggregated data from two tertiary hospitals in Kota Bharu and Johor Bahru with a waiver of patient consent after approval by their respective research ethics boards. These two districts rank in Malaysia’s top five most populous districts, with 1,379 and 1,608 inhabitants per square kilometre, respectively [10]. Both districts have international points of entry; Johor Bahru, in peninsular Malaysia’s south, is connected to Singapore by a bridge, whilst Kota Bharu, in the northeast, is bordered to the north by Thailand. More than 25% of the population of people in these districts is under 18 years old. The study involves 264 weeks (five years) of secondary data. We divided the COVID-19 timeline in Malaysia with the declaration of the first MCO on March 18, 2020 (week 12 of 2020) and the termination of the MCO on January 3, 2022 (week 1 of 2022) as the pivotal weeks. Hence, three study periods were defined: the pre-MCO period between March 17, 2017, and March 17, 2020 (week 11 2017 to week 11 2020), the MCO period between March 18, 2020, and January 2, 2022 (week 12 2020 to week 52 2021) and the post-MCO period between January 3, 2022, and March 17, 2022 (week 1 2022 to week 12 2022).

Participants and data source

Patient data were extracted from the electronic medical records of each hospital. Participants included all paediatric patients below 18 years old at the time of the visit and registered in the ED of the respective hospitals, with the exclusion of those who absconded before medical consultation, babies born before arrival, those who came for a scheduled review, test, screening or procedure only, and cases referred from other hospitals. Revisit cases within 24 hours were also excluded to control for admission bias due to local hospital policy requiring all paediatric revisits within 24 hours to be admitted for observation.

Data collection

The primary outcome was the number of paediatric ED visits per week. Three secondary outcomes were further examined: the triage category, visit outcome and ED discharge diagnosis. Trained paramedics categorised the triage upon initial assessment of the patients based on a colour-coded system in which green indicates non-urgent cases, yellow indicates urgent cases and red indicates emergent or life-threatening cases. Meanwhile, visit outcomes referred to discharge, including discharge against medical advice; admission, including admission transfer to other hospitals; and death. Finally, ED discharge diagnoses were classified using the assigned visit International Classification of Disease version 10 (ICD-10) code diagnosed by the attending medical doctor or emergency physician.

Statistical analysis

We used a time series design to enable a longitudinal comparison of outcomes of interest between the exposure (MCO/post-MCO) and control period (pre-MCO). A descriptive analysis and time series graph was plotted to analyse the primary outcome of the total number of paediatric ED visits per week.

For the outcomes of the triage category, visit outcome, and ED discharge diagnosis, we investigated the total weekly number of events and their relative proportion of all ED visits. A Welch t-test was used to compare the weekly mean number of paediatric ED visits between the three study periods considering the unequal lengths of the periods [11]. Multinomial logistic regressions were conducted to compare the odds ratios (ORs) of these events occurring in the MCO and post-MCO period relative to the pre-MCO period. The day of the year was included to control for temporal variation, whereas the hospitals were included to control for spatial variation, as shown in the following equation [12], where x is the outcome of interest:

$$Period \sim x + day of year + hospital.$$

Changepoint analysis using the EnvCpt package version 1.1.3 of the R statistical computing software version 4.2.2 (R Foundation for Statistical Computing, Vienna, Austria) of all outcomes was then conducted to identify if, and where, an abrupt change has occurred within the time series. The data were modelled using a Poisson distribution with no maximum number of changepoints set in the full range. The Pruned Exact Linear Time (PELT) method with the modified Bayesian information criterion (BIC) penalty version was used to identify the changepoints. The EnvCpt package compares 12 models, and the most parsimonious model with the minimum number of BIC was selected.

## Results

A total of 175,737 visits were recorded over the five years. There is an approximately equal distribution of visits between the two study areas (Kota Bharu: 43.19%, Johor Bahru: 56.81%), whilst males are predominant (male: 56.83%, female: 43.17%). More than half of the visits consisted of children below five years old (56.4%), and Malays made up more than 80% of the visits, reflecting the districts’ population demography (Table 1).

**Table 1:** Demographic characteristics of paediatric patients visiting the emergency department from week 11 2017 to week 12 2022

Variables	Total (N=175,737)		Hospital			
			Kota Bharu (n=75,907)		Johor Bahru (n=99,830)	
	Number	%	Number	%	Number	%
Age (years)						
<5	99,094	56.4	38,779	51.1	60,315	60.4
5-12	48,108	27.4	23,374	30.8	24,734	24.8
>12	28,535	16.2	13,754	18.1	14,781	14.8
Gender						
Female	75,878	43.2	33,157	43.7	42,721	42.8
Male	99,859	56.8	42,750	56.3	57,109	57.2
Ethnicity						
Malay	153,165	87.0	74,392	98.0	78.773	78.9
Chinese	10,264	5.8	1,110	1.46	9,154	9.17
Indian	5,725	3.3	91	0.12	5,634	5.64
Other	6,583	3.7	314	0.41	6,269	6.28

The total number of paediatric emergency department visits experienced a steep decline between week 5 2020 and week 10 2020 (Figure 1). There were two visible peaks during the MCO period: between week 30 2020 and week 40 2020, and between week 12 2021 and week 17 2021. A third peak occurred during the transition from MCO to the post-MCO period from week 50 2021 to week 4 2022. A 57.57% reduction (p<0.00) in the average number of paediatric ED visits per week was observed during the MCO period compared to the pre-MCO period, whilst a 34.07% (p<0.00) decrease in average weekly paediatric ED visits from the baseline is observed after the termination of the MCO. Two changepoints were identified for the total number of paediatric ED visits at week 9 2020 and week 50, three weeks before the start and termination of the MCO.

**Figure 1:** Trend of weekly paediatric emergency department visits in two tertiary hospitals in Malaysia in the three periods of pre-MCO, MCO and post-MCO and the circulating COVID-19 variants Emergence of new COVID-19 variants circulating within the community MCO: Movement Control Order, COVID-19: coronavirus disease 2019

Emergency department triage category

When compared to the pre-MCO period, the average weekly number of paediatric visits decreased across all triage categories, with the green category experiencing the largest decline (-59.71%, p<0.00) (Table 2). In contrast to the overall decrease, the weekly average of the red triage category post-MCO shows a substantial rise from the pre-MCO period (75.48%, p<0.00). Despite the overall decline, more paediatric ED patients are presenting with urgent or emergent conditions than non-urgent conditions in comparison to the pre-MCO period. The odds of paediatric ED patients being triaged in the yellow (OR: 1.23, 95% CI: 1.20-1.28, p<0.00) or red (OR: 1.79, 95% CI: 1.69-1.90, p<0.00) categories are greater in the MCO period, whereas the odds of paediatric ED patients being triaged in the red category are highest during the post-MCO period (OR: 1.79, 95% CI: 1.69-1.90, p<0.00).

**Table 2:** Changes in the paediatric emergency department visits by triage category and visit outcomes in the MCO period and post-MCO period compared with the pre-MCO period MCO: Movement Control Order, df: Degree of freedom, t: Welch test statistic, d: Cohen’s d, OR: odds ratio, CI: confidence interval

Variable	Period	Number of visits					Proportion of visits		
		% of baseline	df	t	p-value	d	OR	95% CI	p-value
Triage category									
Green	MCO	-59.71	244.7	35.20	<0.00	4.38	0.11	0.11-0.12	<0.00
	Post-MCO	-43.60	12.3	8.20	<0.00	2.58	0.41	0.40-0.44	<0.00
Yellow	MCO	-53.31	234.3	19.20	<0.00	2.42	1.23	1.20-1.28	<0.00
	Post-MCO	-6.18	12.1	0.69	0.50	0.23	1.65	1.54-1.76	<0.00
Red	MCO	-20.43	150.7	4.40	<0.00	0.60	1.79	1.69-1.90	<0.00
	Post-MCO	75.48	11.2	-3.48	<0.00	1.33	3.36	3.00-3.77	<0.00
Visit outcome									
Discharged	MCO	-61.92	247.9	36.10	<0.00	4.46	0.61	0.60-0.63	<0.00
	Post-MCO	-36.69	12.1	6.06	<0.00	1.98	0.76	0.71-0.81	<0.00
Admitted	MCO	-36.17	149.7	13.31	<0.00	1.80	0.19	0.18-0.19	<0.00
	Post-MCO	-21.08	11.7	2.85	0.03	0.99	0.61	0.57-0.66	<0.00
Death	MCO	-16.27	209.5	0.93	0.35	0.12	1.24	0.86-1.80	0.25
	Post-MCO	-38.44	13.4	1.05	0.31	0.29	1.08	1.06-1.09	<0.00

Other than paediatric patients in the yellow triage categories post-MCO and red triage categories during the MCO, a large effect size of more than 0.8 is evident in the total number of patients compared to the pre-MCO period. According to their triage categories, this suggests that there was a greater than 79% difference in the weekly average of patients between the MCO and post-MCO periods compared to the post-MCO period. The difference between the green categories during the MCO period (d=4.38) and post-MCO period (d=2.58) compared to the pre-MCO period has the biggest effect size.

The models with changepoints in the mean and the second-order autocorrelation process observed abrupt changes in the trend of the triage categories. Ten weeks before the MCO began, in week 2 of 2020, the first shift was noted in the green triage category (Figure 2a). An abrupt decrease followed this in the yellow and red triage category trend before the MCO (Figure 2b and Figure 2c). Another changepoint was observed in weeks 51 and 43 of 2021 for the yellow and red triage categories, respectively.

**Figure 2:** Detected changepoints in the trend of paediatric emergency department visits by triage categories based on the model with minimum BIC value The vertical blue lines indicate influential changepoints within the time series. The pink shaded area indicates the Movement Control Order period in Malaysia. ED: emergency department, BIC: Bayesian information criterion

Emergency department visit outcome

Both the MCO and post-MCO periods observed a marked decline in the average number of paediatric patients discharged from the emergency department or admitted to the hospital per week in contrast to the pre-MCO period (Table 2). The biggest drop is seen in the average weekly number of paediatric patients discharged during the MCO period (-61.92%, p<0.00). During the MCO and post-MCO periods, paediatric patients who attend the ED have reduced odds of being discharged or admitted. On the other hand, the odds that a child will die after visiting the ED in the post-MCO period is relatively similar to the pre-pandemic period (OR: 1.08, 95% CI: 1.06-1.09, p<0.00).

A substantial effect size was reported for both discharged and admitted visit outcomes during the MCO and post-MCO periods. The difference in the average weekly number of patients discharged during the MCO period (d=4.46), with a 99.9% difference from the baseline, has the biggest effect size. The average number of patients admitted weekly during the MCO (d=1.80) and post-MCO (d=0.99) differed from baseline by 79%-96%.

A changepoint was seen for both the discharged and admitted outcomes in week 9 of 2020, three weeks before the MCO began (Figure 3a and Figure 3b). Although hospital admissions fluctuated after the MCO started, no influential changepoints were observed. In contrast, a shift leading to an increased number of patients discharged from the ED was seen in week 50 of 2021. No changepoints were identified in the trend for paediatric patients who visited the ED resulting in death (Figure 3c).

**Figure 3:** Detected changepoints in the trend of paediatric emergency department visit outcomes based on models selected with minimum BIC value The vertical blue lines indicate influential changepoints within the time series. The pink shaded area indicates the Movement Control Order period in Malaysia. ED: emergency department, BIC: Bayesian information criterion

Emergency department discharge diagnosis

Due to no diagnosis (28,794 cases, 15.2%) and outliers from the chemical spill incident in Johor Bahru (294 cases, 0.2%), 29,088 cases were excluded from this analysis. The respiratory system, fever or other infectious diseases, burn or trauma and the gastrointestinal system remain the top diagnoses across the three periods of COVID-19. We also noticed that the top 10 diagnoses in the post-MCO period no longer included diagnoses for perinatal disorders, such as neonatal jaundice and neonatal presumptive sepsis, as illustrated in Figure 4.

**Figure 4:** Ranking of emergency department-related diagnosis for paediatric patients during the pre-MCO, MCO and post-MCO periods MCO: Movement Control Order

Further analysis of the top five diagnoses reveals a general decrease in average weekly visits for these conditions over the MCO and post-MCO periods compared to the pre-MCO period, with the most significant decline being the diagnosis for conditions originating in the perinatal period after the termination of the MCO (-94.55%, p<0.00) (Table 3). A large effect size was seen for all five diagnoses compared to the pre-MCO period, with Cohen’s d values ranging from 0.90 to 4.80. Compared to the other four most common diagnoses, paediatric patients who attend the ED during the MCO period have the lowest odds of receiving a respiratory diagnosis (OR: 0.53, 95% CI: 0.51-0.56, p=0.00). Whilst in the post-MCO period, paediatric patients who attend the ED have the lowest odds of having a condition originating in the perinatal period (OR: 0.07, 95% CI: 0.05-0.10, p<0.00).

**Table 3:** Changes in the paediatric emergency department visits of the top five diagnoses in the MCO and post-MCO periods compared with the pre-MCO period MCO: Movement Control Order, df: degree of freedom, t: Welch test statistic, d: Cohen’s d, OR: odds ratio, CI: confidence interval

Diagnosis	Period	Number of visits					Proportion of visits		
		% of baseline	df	t	p-value	d	OR	95% CI	p-value
Respiratory system	MCO	-70.25	231.3	28.69	<0.00	3.63	0.53	0.51-0.56	0.00
	Post-MCO	-22.15	12.0	2.74	0.01	0.90	1.00	0.93-1.08	0.91
Fever or other infectious diseases	MCO	-62.42	249.6	20.65	<0.00	2.52	0.59	0.56-0.62	0.00
	Post-MCO	-40.07	15.8	6.75	<0.00	1.59	0.66	0.61-0.72	0.00
Burn or trauma	MCO	-39.27	190.3	17.16	<0.00	2.24	1.02	0.97-1.06	0.47
	Post-MCO	-38.09	12.2	6.28	<0.00	2.02	0.85	0.77-0.93	0.00
Gastrointestinal system	MCO	-59.26	249.3	28.19	<0.00	3.47	0.69	0.65-0.72	0.00
	Post-MCO	-33.82	12.0	4.25	0.00	1.41	0.88	0.80-0.97	0.01
Conditions originating in the perinatal period	MCO	-36.35	169.2	8.93	<0.00	1.19	0.97	0.91-1.13	0.34
	Post-MCO	-94.55	93.1	36.49	<0.00	4.80	0.07	0.05-0.10	<0.00

Our findings show that the number of paediatric ED patients being diagnosed with fever or other infectious diseases had drastically increased 12 weeks before the start of the MCO at week 51 2019 and peaked in week 4 2020, before rapidly declining until two weeks after the MCO (week 14 2020) (Figure 5b). In contrast, the changepoints in the pre-MCO period for paediatric respiratory and gastrointestinal cases marked a decline in the number of cases for these conditions (Figure 5a and Figure 5d). During the MCO period, the changepoints indicated a sudden rise in the number of cases for the diagnosis of respiratory, fever or other infectious diseases, or gastrointestinal cases. Contrarily, the diagnosis of complications originating from the perinatal period experienced an abrupt decrease in trend in week 29 2021 (Figure 5e). No influential changepoints were identified in the trend for the diagnosis of burns and trauma (Figure 5c).

**Figure 5:** Detected changepoints in the trend of the top five diagnoses of paediatric patients visiting the emergency department based on models selected with minimum BIC value The vertical blue lines indicate influential changepoints within the time series. The pink shaded area indicates the Movement Control Order period in Malaysia. ED: emergency department, BIC: Bayesian information criterion

## Discussion

In this multicentre study in Malaysia, the average number of weekly paediatric ED visits declined by 57.57% after MCO implementation, with a contralateral rise in the odds of paediatric patients triaged as yellow and red categories. Several possible factors can explain the decrease in paediatric ED visits. The first factor was speculated to be driven by the healthcare system reform. During the MCO, dynamic changes in healthcare service delivery were made. The study sites were amongst the selected tertiary hospitals that were gazetted as COVID-19 hospitals, leading to structural reorganisation in the emergency department. Amongst them, non-urgent paediatric patients, including minor cases of upper respiratory tract infections or fever, were encouraged to seek medical attention from public or private health clinics to segregate patients based on their risk for COVID-19 [13].

Parental concern was another possible factor for the decline in paediatric ED utilisation. Earlier epidemics have reported parental fear of infection from the ED as a deterring factor for paediatric ED visits [14]. Although parents seeking medical treatment for their children from virtual consultations or private practices has become an alternative, a potential increase in the delayed presentation of paediatric patients may explain the rise in the yellow and red triage categories of cases [15]. This, however, is beyond the scope of this study.

We expected an increase in the proportion of admission during the MCO period considering the higher proportion of urgent (yellow triage category) and emergent (red triage category) patients, as evidenced in Korea [9] and Canada [8]. However, this study surprisingly shows that both proportions of discharged and admitted paediatric patients decreased during the MCO and post-MCO periods. We speculated that allocating COVID-19 dedicated wards in our hospitals has reduced the number of available hospital beds. Thus, stricter admission criteria were practised in the emergency department. Concurrently, COVID-19 quarantine and treatment centres were set up throughout the country to offload hospital patient care burden. Asymptomatic or mildly symptomatic and stable COVID-19 patients diagnosed in the ED were discharged from the ED’s system and were admitted to these centres.

The international travel ban in Malaysia was lifted in phases starting from week 41 of 2021. A surge in international travel was observed with a subsequent increase in the number of imported COVID-19 cases detected, especially amongst travellers to Mecca for the pilgrimage [16]. Consequently, the COVID-19 Omicron variant replaced the community’s circulating variant. With the shift from Beta, Alpha and Delta variants of the COVID-19 virus, we observe peaks in paediatric ED visits despite an overall decline in the number of visits. The high infectivity of the Omicron variant had caused an unprecedented surge in the number of paediatric visits. A similar observation was reported by Iijimaet al. [17] in Japan and Taytard et al. [18] in France, thus highlighting the importance of disease and laboratory surveillance.

Malaysia had robustly introduced a new norm of dos and don’ts for infection control within the community during the pandemic. The ‘dos’ include wearing face masks in public, frequently washing one’s hands with water and soap or using hand sanitiser and obeying the warnings by the Ministry of Health, such as staying at home. The ‘don’ts’ include avoiding crowded areas, conversing close to others and being in confined spaces. Whilst the initial intention of these recommendations was to curb the transmission of COVID-19 via air droplets, a cascading positive effect of preventing other diseases was observed [19]. The decline in fever and other infectious diseases during the MCO period substantiates this observation. The variance for fever and other infectious disease cases was seen to revert to the pre-MCO era as the school reopens in phases beginning in week 40 2020, albeit no influential changepoint was detected. It is theorised that difficulty enforcing the new standard amongst school-going children may be the cause [20].

Furthermore, the decline in the conditions originating from the perinatal period is postulated to reflect the overall decrease in live births in Malaysia. The argument is congruent with a report stating a 3.6% drop in live births from 15 in 2019 to 14.4 in 2020 for every 1,000 people [21]. This trend differs from Thailand, Peru and the USA, which reported a slight decline in births at the beginning of 2021 before experiencing a rebound to the pre-pandemic trend, possibly due to delayed birth registration [22]. The current findings were instead similar to the situation in Italy, where the authors speculated that the stringent and prolonged lockdown had adversely affected the mental health and subsequent sexual drive of their population [23]. Furthermore, the fear of economic instability due to reduced earnings may have been the contributing factor [24].

Limitations

Four limitations must be highlighted in the current study. First, although when planned, a prolonged study period seemed ideal considering the protracted and dynamic nature of the COVID-19 pandemic, in retrospect, the unequal length of each period could have been adjusted through truncation or implementation of an interrupted time series. However, this is at the expense of potentially wasting useful information. Second, we did not obtain primary information from the patients or their caregivers. Therefore, we were unable to glean insight into parental motivation on the timing of seeking emergency medical treatment as well as the respective socioeconomic impact that influences their accessibility or affordability to seek treatment. Third, we were also unable to gain access to data from the private sector, thus limiting the generalizability of our study. Finally, there needed to be more clarity in the diagnostic terms used by the two hospitals. Although we have coded the diagnoses based on the ICD-10 codes to the best of our ability, considering the volume of paediatric ED visits in Malaysia, expanding the study to other centres may benefit from a prospective study with predetermined codes for a more accurate representation of diseases.

## Conclusions

The implementation of the Movement Control Order in Malaysia was associated with a profound decrease in the number of paediatric emergency department visits in public tertiary hospitals and emphasised the importance of disease and laboratory surveillance. The incongruent decline in the proportion of admission, as opposed to an increased proportion of the yellow and red triage cases, highlights the potential effects of the healthcare system reform and the socioeconomic impact of the pandemic on paediatric ED utilisation. Concurrently, the trend of ED discharge diagnoses provides evidence of the nation’s effectiveness in controlling disease transmission within the community.
